# Multi-Layer Perceptron Classifier with the Proposed Combined Feature Vector of 3D CNN Features and Lung Radiomics Features for COPD Stage Classification

**DOI:** 10.1155/2023/3715603

**Published:** 2023-11-03

**Authors:** Yingjian Yang, Nanrong Zeng, Ziran Chen, Wei Li, Yingwei Guo, Shicong Wang, Wenxin Duan, Yang Liu, Rongchang Chen, Yan Kang

**Affiliations:** ^1^College of Medicine and Biological Information Engineering, Northeastern University, Shenyang 110169, China; ^2^College of Health Science and Environmental Engineering, Shenzhen Technology University, Shenzhen 518118, China; ^3^School of Applied Technology, Shenzhen University, Shenzhen 518060, China; ^4^Shenzhen Institute of Respiratory Diseases, Shenzhen People's Hospital, Shenzhen 518001, China; ^5^The Second Clinical Medical College, Jinan University 518001, Guangzhou, China; ^6^The First Affiliated Hospital, Southern University of Science and Technology 518001, Shenzhen, China; ^7^Engineering Research Centre of Medical Imaging and Intelligent Analysis, Ministry of Education, Shenyang 110169, China

## Abstract

Computed tomography (CT) has been regarded as the most effective modality for characterizing and quantifying chronic obstructive pulmonary disease (COPD). Therefore, chest CT images should provide more information for COPD diagnosis, such as COPD stage classification. This paper proposes a features combination strategy by concatenating three-dimension (3D) CNN features and lung radiomics features for COPD stage classification based on the multi-layer perceptron (MLP) classifier. First, 465 sets of chest HRCT images are automatically segmented by a trained ResU-Net, obtaining the lung images with the Hounsfield unit. Second, the 3D CNN features are extracted from the lung region images based on a truncated transfer learning strategy. Then, the lung radiomics features are extracted from the lung region images by PyRadiomics. Third, the MLP classifier with the best classification performance is determined by the 3D CNN features and the lung radiomics features. Finally, the proposed combined feature vector is used to improve the MLP classifier's performance. The results show that compared with CNN models and other ML classifiers, the MLP classifier with the best classification performance is determined. The MLP classifier with the proposed combined feature vector has achieved accuracy, mean precision, mean recall, mean *F*1-score, and AUC of 0.879, 0.879, 0.879, 0.875, and 0.971, respectively. Compared to the MLP classifier with the 3D CNN features selected by Lasso, our method based on the MLP classifier has improved the classification performance by 5.8% (accuracy), 5.3% (mean precision), 5.8% (mean recall), 5.4% (mean *F*1-score), and 2.5% (AUC). Compared to the MLP classifier with lung radiomics features selected by Lasso, our method based on the MLP classifier has improved the classification performance by 5.0% (accuracy), 5.1% (mean precision), 5.0% (mean recall), 5.1% (mean *F*1-score), and 2.1% (AUC). Therefore, it is concluded that our method is effective in improving the classification performance for COPD stage classification.

## 1. Introduction

Chronic obstructive pulmonary disease (COPD) is a common and non-infectious lung disease characterized by persistent airflow limitation [1–3]. Because of this characterization, the COPD stage is diagnosed from stage 0 to IV according to Global Initiative for Chronic Obstructive Lung Disease (GOLD) criteria accepted by the American Thoracic Society and the European Respiratory Society [4]. GOLD is examined by the pulmonary function test (PFT) and diagnosed by the forced expiratory volume in 1 second/forced vital capacity (FEV1/FVC) and FEV1% predicted [1, 2]. PFT can explain the impact on symptoms and life quality of COPD patients [5, 6], but it cannot reflect the change of the lung tissue in COPD patients with the COPD stage evolution. PFT changes from normal to abnormal occur when lung tissue is destroyed to a certain extent. Therefore, the PFT makes it challenging to identify the etiology of COPD.

Compared with the GOLD criteria and other imaging equipment, computed tomography (CT) has been regarded as the most effective modality for characterizing and quantifying COPD [7]. Compared with PFT, chest CT images can indicate that the patients have suffered from mild lobular central emphysema and decreased exercise tolerance in smokers without airflow limitation [8]. In addition, the chest CT images are also used to quantitatively analyze the bronchial, airway disease, emphysema, and vascular for COPD patients [7]. However, automatic multi-classification based on convolutional neural networks (CNNs) using chest CT images remains a challenging task for the COPD stage. One main reason is that the number of medical images is limited compared to natural images. In particular, few people seek medical treatment in the early stage of COPD and undergo CT scans simultaneously. Transfer learning [9] may solve the above problems. Since radiomics was proposed to mine more information from medical images using advanced feature analysis in 2007 [10], it has been widely used to analyze lung disease imaging [11–15]. However, radiomics features are extracted from medical images by specific calculation equations, preset types of images, and preset classes, limiting the forms of radiomics features. Some deep features from CNN (CNN features) are also needed to improve the classifier's performance in multi-classification. CNN features extracted from medical images will make up for the limitations of radiomics features.

Radiomics features in COPD develop slower than those in other lung diseases, such as lung cancer and pulmonary nodules. Until 2020, reference [16] points out that radiomics features in COPD have not been extensively investigated yet. Nevertheless, there are potential applications of radiomics features in COPD for the diagnosis, treatment, and follow-up of COPD and future directions [16]. A critical reason limiting the development of radiomics features in COPD is its diffuse distribution in the lung. At the same time, radiomics features need to be extracted from the region of interest (ROI) of the chest CT images. However, the diffuse distribution of COPD makes it difficult to determine ROI. COPD results from the joint action of the peripheral airway, pulmonary parenchyma, and pulmonary vessels [17–19]. Thus, the peripheral airway, pulmonary parenchyma, and pulmonary vessels as ROI to extracting lung radiomics features are reasonable for COPD stage classification.

Currently, radiomics features also have been used in COPD for survival prediction [20, 21], COPD presence prediction [22], COPD exacerbations [23], COPD early decision [4], and analysis of COPD and resting heart rate [3]. However, as mentioned above, lung radiomics features have not been applied in the COPD stage classification. On the other hand, radiomics based on machine learning (ML) and chest CT images based on CNN have been widely and respectively used in COPD and its evaluation. However, the advantages of radiomics based on machine learning and medical images based on CNN need to be further integrated to improve the performance of COPD stage classification. Therefore, this paper proposes a feature combination strategy by concatenating three-dimension (3D) CNN features and lung radiomics features for COPD stage classification based on the multi-layer perceptron (MLP) classifier. Our contributions in this paper are briefly described as follows. (1) MLP classifier with the best classification performances is determined in the ML classifier for 3D CNN features or lung radiomics features. (2) Truncated transfer learning is proposed from the excellent segmentation model for generating nonlinear 3D CNN features. (3) The proposed feature combination strategy by concatenating 3D CNN features and lung radiomics features effectively improves the MLP classifier's performance.

## 2. Materials and Methods

### 2.1. Materials

The participants are enrolled by the national clinical research center of respiratory diseases, China, from May 25, 2009, to January 11, 2011. Finally, 465 Chinese subjects participated in the study after being strictly selected by the inclusion and exclusion criteria [24]. The 465 subjects underwent chest HRCT scans at the full inspiration state. In addition, the 465 subjects also underwent the PFT, and the COPD stage of each subject is diagnosed by PFT in Global Initiative for Chronic Obstructive Lung Disease (GOLD) criteria 2008 accepted by the American Thoracic Society and the European Respiratory Society.

Figure 1 shows the COPD stage distribution of the subjects in this study. There are 129, 108, 121, and 107 subjects in each COPD stage (GOLD 0, GOLD I, GOLD II, GOLD III, and GOLD IV). This study was approved by the ethics committee of the national clinical research center for respiratory diseases in China. In addition, all 465 subjects have been provided written informed consent to the first affiliated hospital of Guangzhou medical university before chest HRCT scans and PFT. Refer to our previous study [4] for a more detailed description of the materials.

### 2.2. Methods

Figure 2 shows the proposed method in this study. The main idea of the proposed method proposed in this paper is to combine 3D CNN features and lung radiomics features for COPD stage classification. When generating the 3D CNN features, we adopt a truncated transfer learning strategy that only intercepts the encoder backbone of the pretrained Med3d [25].

#### 2.2.1. Lung Radiomics Features Extraction

First, 465 sets of chest HRCT images are automatically segmented by a trained ResU-Net [26], obtaining 465 sets of lung images with the Hounsfield unit (Hu) [27]. The lung images include the peripheral airway, pulmonary parenchyma, and pulmonary vessels. The architecture of the ResU-Net has been described in detail in our previous study [28]. Then, lung radiomics features of 465 subjects are extracted from the lung images by PyRadiomics [29]. Refer to our previous study [4] for a more detailed description of the lung radiomics feature extraction.

#### 2.2.2. 3D CNN Feature Extraction

A truncated transfer learning strategy is proposed to extract the 3D CNN features based on the pretrained Med3d [25]. Med3d, a heterogeneous 3D network, is used to extract general medical 3D features by building a 3DSeg-8 dataset with diverse modalities, target organs, and pathologies. Thus, we only transfer the encoder backbone of the pretrained Med3d (3D ResNet10) for generating the 3D CNN features, as shown in Figure 2(a).

Figure 2(b) shows that the 465 sets of lung images with Hu are input to the transferring encoder backbone, generating CNN feature vectors in detail. First, the lung images (512 × 512 × *N*) are cropped into the size 280 × 400 × *N*′, retaining the lung region. The non-lung images are also deleted, so *N* changes into *N*′ (*N*′ < *N*). Second, the cropped lung images are preprocessed by the method in reference [25], normalizing the lung region and generating random values outside the lung region in accordance with Gaussian distribution. Equation (1) shows the mathematical form of normalization:

(1) $$\begin{array}{c} x^{\prime }=\frac{x-\bar{x}}{\sigma }, \end{array}$$

where *x* is the value of the lung region, $\bar{x}$ is the mean value of the lung region, and *σ* is the mean square deviation of the lung region.

Third, the CNN feature maps (512 × 35 × 50 × 75) are generated by the cropped and preprocessed lung images (1 × 280 × 400 × N′) and the pretrained Med3d. Last, higher-order CNN feature maps (512 × 3 × 3 × 3) need to be extracted from the CNN feature maps (512 × 35 × 50 × 75) by 3D average pooling. Then, the higher-order CNN feature maps (512 × 3 × 3 × 3) are flattened into the CNN feature vector. Finally, each CNN feature vector (per subject) includes 13824 3D CNN features (512 × 3 × 3 × 3 = 13824).

#### 2.2.3. Combined Feature Vector for COPD Classification

Figure 2(c) shows that the combined feature vector is generated by concatenating the CNN feature vector and the radiomics feature vector. First, the CNN feature vector (13824) and the radiomics feature vector (1316) are selected by the least absolute shrinkage and selection operator (Lasso) [30], respectively. After Lasso, the number of the selected CNN feature vector and the selected radiomics feature vector is 60 and 106, respectively. A standard python package LassoCV, with tenfold cross-validation, is performed in this paper. Equation (2) shows the mathematical form of Lasso [4]:

(2) $$\begin{array}{c} A\leftarrow \;\arg\;\min\left\{\overset{n}{\underset{i=1}{\sum }}{\left(y_{i}-\beta_{0}-\overset{p}{\underset{j=1}{\sum }}\beta_{j}x_{\text{ij}}\right)}^{2}+\lambda \overset{p}{\underset{j=0}{\sum }}\left|\beta_{j}\right|\right\}, \end{array}$$

where matrix *A* denotes the selected lung radiomics feature. *x*_ij_ denotes the lung radiomics features (the independent variable). *y*_*i*_ denotes the COPD stage (the independent variable). *λ* denotes the penalty parameter (*λ* ≥ 0). *β*_*j*_ denotes the regression coefficient, *i* ∈ [1, *n*], and *j* ∈ [0, *p*].

Second, the combined feature vector is generated by concatenating the selected CNN feature vector and the selected radiomics feature vector. Finally, the combined feature vector is the size 1 × 166 per subject.  Figure 2(d) shows that MLP [31, 32] with the combined feature vector is used to classify the COPD stage in this paper.

#### 2.2.4. Experiments and Evaluation Metrics

Our proposed method uses the combined feature vector of 3D CNN features and lung radiomics features for COPD stage classification based on the MLP classifier. Our experiment includes five experiments in this section to verify the effectiveness of our proposed method.

Figure 3 shows the experimental design in this paper. End-to-end CNN models based on parenchyma images are used for COPD stage classification in experiments 1-2. Specifically, two classic CNN models, DenseNet and GoogLeNet, based on parenchyma images, are adopted to compare the classification performance of the six different ML classifiers. The classification performance of DenseNet and GoogleNet has been evaluated by our previous study [33], which achieved the best classification performance for image classification. Furthermore, compared with experiment 1, multiple-instance learning (MIL) [34], a form of weakly supervised learning, is applied in experiment 2. Meanwhile, different ML classifiers based on different feature vectors are also used for COPD stage classification in experiments 3–5.

Specifically, the training parameters of 2D DenseNet and 3D DenseNet are set: 20/2 (batch size (2D/3D)), 512 × 512/512 × 512 × 20^*∗*^ (input size (2D/3D)), 50/50 (epoch (2D/3D)), and 0.5/0.2 (drop rate (2D/3D)) in experiment 1. The training parameters of 2D GoogleNet and 3D GoogleNet are set: 16/2 (batch size (2D/3D)), 512 × 512/512 × 512 × 20^*∗*^ (input size (2D/3D)), 50/50 (epoch (2D/3D)), and 0.2/0.2 (drop rate (2D/3D)) in experiment 1. ^*∗*^MIL: each case (a set of chest HRCT images) was equally divided into 20 segments, with one slice taken equidistantly to obtain 20 slices in each case. The training parameters of 2D DenseNet with MIL (2D DenseNet_MIL) and 3D DenseNet with MIL (3D DenseNet_MIL) are set: 16/2 (batch size (2D/3D)), 512 × 512^*∗∗*^/512 × 512 ×  × 512 × 16^*∗∗∗*^ (input size (2D/3D)), 50/50 (epoch (2D/3D)), and 0.5/0.2 (drop rate (2D/3D)) in experiment 2. The training parameters of 2D GoogleNet with MIL (2D GoogleNet_MIL) and 3D GoogleNet with MIL (3D GoogleNet_MIL) are set: 16/2 (batch size (2D/3D)), 512 × 512∗∗/512 × 512 × 16^*∗∗∗*^ (input size (2D/3D)), 50/50 (epoch (2D/3D)), and 0.2/0.2 (drop rate (2D/3D)) in experiment 2. ^*∗∗*^MIL: each case was equally divided into 10 bags, with one slice taken randomly to obtain 10 slices in each case. ^*∗∗∗*^MIL: each case was equally divided into 16 bags, with one slice taken equidistantly to obtain 16 slices in each case.

Specifically, experiments 3–5 are designed to compare the classification performance of the six different classifiers based on the CNN feature vector (13824), radiomics feature vector (1316), their selected feature vector by Lasso, and the proposed combined feature vector (166), respectively. First, based on 3D ResNet10, we use six classic classifiers (SVM [35], MLP, RF [36], LR [37], GB [38], and LDA [39]) to determine the best COPD classification classifier by different feature vectors.  Table 1 reports the six different classifiers with their definitions in this paper. The different feature vectors include the CNN feature vector (13824), CNN feature vector selected by Lasso (60), radiomics feature vector (1316), and radiomics feature vector selected by Lasso (106). The MLP classifier with the best classification performance is determined. Second, we further verify the proposed combined feature vector (166) to improve the MLP classifier's performance. Third, 3D ResNet18 and 3D ResNet34 are also transferred to generate the CNN feature vector, and the 3D ResNet10 is determined as the encoder backbone with the best performance on the MLP classifier. The 465 subjects are divided into the train set (70%) and the test set (30%).  Figure 4 shows the detailed dataset division for training and test set in each COPD stage.

Standard evaluation metrics of the CNN and ML models include the accuracy, precision, recall, *F*1-score, and area under the curve (AUC). The above standard evaluation metrics are defined as in equations (3)–(6). The evaluation metric AUC for multi-classification is calculated by the receiver operating characteristic curve (ROC) [40].

(3) $$\begin{array}{c} \text{Accuracy}=\frac{\text{TP}+\text{TN}}{\text{TP}+\text{TN}+\text{FP}+\text{FN}}, \end{array}$$

(4) $$\begin{array}{c} \text{Precision}=\frac{\text{TP}}{\text{TP}+\text{FP}}, \end{array}$$

(5) $$\begin{array}{c} \text{Recall}=\frac{\text{TP}}{\text{TP}+\text{FN}}, \end{array}$$

(6) $$\begin{array}{c} F1-\text{score}=\frac{2\times \text{Precision}\times \text{Recall}}{\text{Precision}+\text{Recall}}, \end{array}$$

where the true positive (TP) and false positive (FP), respectively, represent the positive and negative samples classified to be positive by the CNN and ML models and the true negative (TN) and false negative (FN), respectively, represent the positive and negative samples classified to be negative by the CNN and ML models.

## 3. Results

This section reports the experimental results, including (1) the classification performance of the parenchyma images based on the DenseNet and GoogleNet; (2) the classification performance of the CNN feature vector and lung radiomics vector based on different classifiers; (3) the MLP classifier's performance with the combined feature vector; and (4) the MLP classifier's performance with combined feature vector based on different 3D ResNet.

### 3.1. The DenseNet and GoogleNet's Performance with Parenchyma Images

This section shows the classification performance of 2D/3D DenseNet, 2D/3D GoogleNet, 2D/3D DenseNet_MIL, and 2D/3D GoogleNet_MIL based on the parenchyma images, respectively.

Figure 5 intuitively shows the AUC of the CNN models by drawing the ROC curves. Tables 2 and 3 report the classification performance of CNN models. Specifically, Table 2 shows that 2D GoogleNet with parenchyma images performs the best in 2D CNN models, achieving 0.550 (accuracy), 0.562 (mean precision), 0.550 (mean recall), 0.553 (mean *F*1-score), and 0.809 (AUC). In addition, Table 3 shows that 3D DenseNet with parenchyma images performs the best in 3D CNN models, achieving 0.579 (accuracy), 0.614(mean precision), 0.579 (mean recall), 0.579 (mean *F*1-score), and 0.787 (AUC).

### 3.2. The Classification Performance of CNN Feature Vector and Lung Radiomics Vector Based on Different Classifiers

This section shows the classification performance of the CNN feature vector (13824), the CNN feature vector selected by Lasso (60), the lung radiomics vector (1316), and the lung radiomics vector selected by Lasso (106) based on different classifiers, respectively.

Figure 6 intuitively shows the AUC of the different classifiers by drawing the ROC curves. Tables 4–7 show that the MLP classifier is the best classifier for COPD stage classification. Specifically, Table 4 reports the classification performance of the different classifiers with the CNN feature vector (13824), respectively. The best classifier is the MLP classifier with 0.793 (accuracy), 0.798 (mean precision), 0.793 (mean recall), 0.790 (mean *F*1-score), and 0.790 (AUC), respectively.  Table 5 reports that the classification performance of the MLP classifier with the CNN feature vector selected by Lasso has improved with 0.821 (accuracy), 0.826 (mean precision), 0.821 (mean recall), 0.821 (mean *F*1-score), and 0.946 (AUC), respectively.  Table 6 reports that the classification performance of the MLP classifier with the radiomics feature vector selected by Lasso has improved with 0.786 (accuracy), 0.784 (mean precision), 0.784 (mean recall), 0.784 (mean *F*1-score), and 0.919 (AUC), respectively.  Table 7 reports that the classification performance of the MLP classifier with the radiomics feature vector selected by Lasso has improved with 0.829 (accuracy), 0.828 (mean precision), 0.829 (mean recall), 0.824 (mean *F*1-score), and 0.950 (AUC), respectively.

Table 5 also reports that Lasso only plays a role in improving the classification performance of the MLP classifier with the CNN feature vector. It does not improve the classification performance of other classifiers with the CNN feature vector. However, Table 7 reports that Lasso does play a role in improving the classification performance of all classifiers with the radiomics feature vector.

### 3.3. The MLP Classifier's Performance with Combined Feature Vectors

The best MLP classifier is determined with the CNN feature vector selected by Lasso (60) or the lung radiomics vector selected by Lasso (106) by Section 3.1. This section shows the classification performance of the MLP classifier with combined feature vectors.

Figure 7 intuitively shows the confusion matrix and ROC curves of the MLP classifier with different feature vectors based on 3D ResNet10. The MLP classifier's performance with different feature vectors reported in Table 8 can be calculated from the confusion matrix. Table 8 reports that the proposed combined feature vectors improve the MLP classifier's performance, achieving 0.879 (accuracy), 0.879 (mean precision), 0.879 (mean recall), 0.875 (mean *F*1-score), and 0.971 (AUC), respectively.

### 3.4. The MLP Classifier's Performance with Combined Feature Vector Based on Different 3D ResNet

The best MLP classifier is determined with the CNN feature vector selected by Lasso (60) or the lung radiomics vector selected by Lasso (106) by Section 3.1. This section shows the classification performance of the MLP classifier with combined feature vectors.

Figure 8 intuitively shows the confusion matrix and ROC curves of the MLP classifier with combined feature vectors based on different 3D ResNet. The MLP classifier's performance with combined feature vectors based on different 3D ResNet reported in Table 7 can be calculated from the confusion matrix.  Table 9 reports that the MLP classifier with combined feature vectors based on 3D ResNet10 achieves the best classification performance.

## 4. Discussion

This paper proposes a features combination strategy by concatenating 3D CNN features and lung radiomics features for COPD stage classification based on the MLP classifier. Three sections are discussed in this section, and we also point out the limitations in this study and the future direction.

First, 2D GoogleNet with parenchyma images performs the best in 2D CNN models. The main reason is that 2D GoogleNet is designed for 2D natural image classification (RGB images). Therefore, it achieves the best classification performance in 2D parenchyma images. Meanwhile, because of the ability to extract interlayer information, 3D DenseNet with parenchyma images performs the best classification in 3D CNN models. However, CNN models with parenchyma images fail to classify the COPD stage. One main reason is that the chest HRCT image cannot fully reflect COPD's characteristics for the CNN models. Specifically, the gold standard of COPD classification is characterized by airflow restriction with a slight difference in the chest HRCT image. The slight difference in COPD is mainly caused by small airway disease with an airway diameter<2 mm [17]. Because of the limitation of HRCT resolution, the above differential features of the small airway will be further blurred in the chest HRCT image. Another reason is that chest HRCT images can reflect the COPD anatomical characteristics, but COPD patients are with high heterogeneity and different phenotypes [1]. The heterogeneity and different phenotypes often result in different features of the chest HRCT images in the same stage. Therefore, it is hard for CNN models to learn specific COPD characteristics, resulting in bad classification performance. At the same time, a set of standard medical images is not as easy to obtain as natural images, and the number of chest HRCT images also restricts CNN models for COPD stage classification. Therefore, compared with CNN models, the ML classifier can realize the COPD stage classification with a small number of samples. This paper determines the MLP classifier with 3D CNN features or lung radiomics features, which performs the best for COPD stage classification. In addition, compared with the convolution layer in the CNN models, the MLP classifier is composed of three full connection layers, which is more efficient and more suitable for modeling long-range dependencies. The MLP classifier also can handle complex nonlinear features and discover dependencies between different input features compared with other classifiers [31, 32]. Meanwhile, the objective evaluation of the COPD stage is only the degree of airflow limitation tested by GOLD criteria [1, 2, 4]. COPD is a heterogeneous disease [41], resulting in differences in features (3D CNN features or lung radiomics features extracted from chest HRCT images) with the same degree of airflow limitation. Therefore, a nonlinear relationship exists between 3D CNN features or lung radiomics features and the COPD stage. Because of this, the MLP classifier is suitable for classifying the COPD stage and has achieved an excellent result in COPD stage classification.

Second, Lasso can improve the classification performance of the MLP classifier with the 3D CNN features and the lung radiomics features. Lasso is often used with survival analysis models to determine variables and eliminate the collinearity problem between variables [30, 42]. The results show that Lasso also can improve the MLP classifier's classification performance by establishing the relationship between the independent variables (3D CNN features or lung radiomics features extracted from chest HRCT images) and dependent variables (the COPD stages). Furthermore, Lasso selects 3D CNN features or lung radiomics features related to COPD stages to reduce the complexity of the MLP classifiers and avoid overfitting [43]. While reducing the complexity of the MLP classifiers, the MLP classifiers can focus on the selected lung radiomics features (the radiomics feature vector selected by Lasso) or the selected 3D CNN features (the CNN feature vector selected by Lasso) and improve the classification performance. From the results of the Lasso, the number of the CNN feature vector selected by Lasso is 60, and that of the radiomics feature vector selected by Lasso is 106. We are surprised that the number of collinearity features in the CNN feature vector is more than that in the radiomics feature vector. This further shows that feature selection of 3D CNN features or the radiomics features is necessary for the COPD stage classification, especially in clinical applications.

Third, the proposed feature combination strategy can further improve the classification performance of the MLP classifier. This paper does not improve the existing classic classifiers and starts with the classification features to enhance the classifier's performance. Many nonlinear classification features, the 3D CNN features, are obtained by a truncated transfer learning strategy. We concatenate the CNN feature vector and the radiomics feature vector for the COPD stage classification, which improves the MLP classifier's performance. The MLP classifier is good at handling complex nonlinear features by itself [31, 32]. Therefore, based on the radiomics feature vector, we add the nonlinear CNN feature vector to the radiomics feature vector, generating a combined feature vector. The combined feature vector with the nonlinear CNN feature vector enhances the MLP classifier's performance. Therefore, this fits the essence of the MLP classifier and is interpretable [44]. The selected encoder backbone of the pretrained Med3D is also directly related to the classification performance. Compared with the MLP classifier with 3D ResNet18 or 3D ResNet34, the MLP classifier with 3D ResNet10 performs the best, consistent with the results of multi-class segmentation task (left lung, right lung, and background) in reference [25].

Finally, this study has some limitations, and we point out the future direction. First, from the materials used in this study, there are not enough cases at the COPD stages III and IV. Second, the existing classic classifiers are not improved. Third, the classification performance of the ML classifier with the 3D CNN features is also limited by the encoder backbone of the pretrained Med3d. In our future work, the recent networks, an auto-metric graph neural network [45], will be further attempted and modified for COPD stage classification based on the 3D CNN features and/or the lung radiomics features.

## 5. Conclusions

This paper proposes a feature combination strategy by concatenating 3D CNN features and lung radiomics features for COPD stage classification based on the MLP classifier. First, the 3D CNN features are extracted from the lung region images based on a truncated transfer learning strategy. Then, the lung radiomics features are extracted from the lung region images by PyRadiomics. Compared with CNN models and other ML classifiers, the MLP classifier with the best classification performance is determined by the 3D CNN features and the lung radiomics features. Lasso plays a role in improving the classification performance of the MLP classifier with the CNN feature vector and the radiomics feature vector. The proposed combined feature vector also improves the MLP classifier's performance. The MLP classifier with the proposed combined feature vector has accuracy, mean precision, mean recall, mean *F*1-score, and AUC of 0.879, 0.879, 0.879, 0.875, and 0.971, respectively. This shows that our method effectively improves the classification performance for COPD stage classification.

## Figures and Tables

**Figure 1:** COPD stage distribution of the subjects in this study.

**Figure 2:** The proposed method in this study. (a) A constructed model of 3D CNN and MLP classifier for COPD stage classification. (b) CNN feature vector is generated by transfer learning from Med3D. (c) The combined feature vector is generated by concatenating the CNN feature vector and the radiomics feature vector. (d) The combined feature vector is used to classify the COPD stage based on MLP classifier.

**Figure 3:** Experimental design in this paper.

**Figure 4:** Dataset division in this paper. (a) Training set. (b) Test set.

**Figure 5:** The ROC curves of the CNN model's performance with parenchyma images. (a) The ROC curves of the 2D/3D DenseNet and 2D/3D GoogleNet. (b) The ROC curves of the 2D/3D DenseNet_MIL and 2D/3D GoogleNet_MIL.

**Figure 6:** The ROC curves of the CNN feature vector and lung radiomics vector are based on different classifiers. (a) The ROC curves of the CNN feature vector (13824). (b) The ROC curves of the CNN feature vector selected by Lasso (60). (c) The ROC curves of the lung radiomics vector (1316). (d) The ROC curves of the lung radiomics vector selected by Lasso (106).

**Figure 7:** The confusion matrix and ROC curves of the MLP classifier with different feature vectors based on 3D ResNet10. (a) The confusion matrix of the MLP classifier with CNN feature vector selected by Lasso (60). (b) The confusion matrix of the MLP classifier with radiomics feature vector selected by Lasso (106). (c) The confusion matrix of the MLP classifier with combined feature vector (166). (d) The ROC curves of the MLP classifier with these feature vectors.

**Figure 8:** The confusion matrix and ROC curves of the MLP classifier with combined feature vectors based on different 3D ResNet. (a) The confusion matrix of the MLP classifier with combined feature vector based on 3D ResNet10. (b) The confusion matrix of the MLP classifier with combined feature vector based on 3D ResNet18. (c) The confusion matrix of the MLP classifier with combined feature vector based on 3D ResNet34. (d) The ROC curves of the MLP classifier with combined feature vectors based on 3D ResNet.

**Table 1:** The different classifiers with their definitions.

Classifier	Model definition in Python 3.6
SVM	SVM sklearn.svm.SVC(kernel = “rbf”,probability = true)
MLP	sklearn.neural_network. MLPClassifier (hidden_layer_sizes = (400, 100), alpha = 0.01, max_iter = 10000)
RF	sklearn.ensemble.RandomForestClassifier(n_estimators = 200)
LR	sklearn.linear_model.logisticRegressionCV(max_iter = 100000, solver = “liblinear”)
GB	sklearn.ensemble.GradientBoostingClassifier()
LDA	sklearn.discriminant_analysis.()

**Table 2:** The 2D DenseNet and 2D GoogleNet's performance with parenchyma images in experiments 1 and 2.

CNN model	Accuracy	Precision (GOLD 0/I/II/III&IV (mean))	Recall (GOLD 0/I/II/III&IV (mean))	*F*1-score (GOLD 0/I/II/III&IV (mean))	AUC
2D DenseNet	0.471	0.800/0.311/0.000/0.720/(0.466)	0.500/0.848/0.000/0.562/(0.471)	0.615/0.455/0.000/0.632/(0.428)	0.730
2D GoogleNet	0.550	0.788/0.419/0.385/0.622/(0.562)	0.650/0.394/0.429/0.719/(0.550)	0.712/0.406/0.405/0.667/(0.553)	0.809
2D DenseNet_MIL	0.493	0.538/0.318/0.333/0.720/(0.477)	0.875/0.424/0.057/0.562/(0.493)	0.667/0.364/0.098/0.632/(0.445)	0.770
2D GoogleNet_MIL	0.414	0.418/0.444/0.368/1.000/(0.545)	0.950/0.121/0.400/0.062/(0.414)	0.580/0.190/0.384/0.118/(0.333)	0.648

**Table 3:** The 3D DenseNet and 3D GoogleNet's performance with parenchyma images in experiments 1 and 2.

CNN model	Accuracy	Precision (GOLD 0/I/II/III&IV (mean))	Recall (GOLD 0/I/II/III&IV (mean))	*F*1-score (GOLD 0/I/II/III&IV (mean))	AUC
3D DenseNet	0.579	0.571/0.429/0.533/0.947/(0.614)	0.800/0.455 0.457/0.562/(0.579)	0.667/0.441/0.492/0.706/(0.579)	0.787
3D GoogleNet	0.393	0.463/0.333/0.279/0.833/(0.471)	0.775/0.061/0.486/0.156/(0.393)	0.579/0.103/0.354/0.263/(0.338)	0.674
3D DenseNet_MIL	0.500	0.500/0.600/0.408/0.900/(0.592)	0.950/0.091/0.571/0.281/(0.500)	0.655/0.158/0.476/0.429/(0.441)	0.741
3D GoogleNet_MIL	0.486	0.471/0.413/0.200/0.789/(0.463)	0.825/0.576/0.029/0.469/(0.486)	0.600/0.481/0.050/0.588/(0.432)	0.746

**Table 4:** The different classifiers' performances based on CNN feature vector (13824) in experiment 3.

Classifier	Accuracy	Precision (GOLD 0/I/II/III&IV (mean))	Recall (GOLD 0/I/II/III&IV (mean))	*F*1-score (GOLD 0/I/II/III&IV (mean))	AUC
SVM	0.629	0.763/0.556/0.514/0.690/(0.635)	0.725/0.606/0.543/0.625/(0.629)	0.744/0.580/0.528/0.656/(0.631)	0.863
MLP	0.793	0.829/0.815/0.806/0.732/(0.798)	0.850/0.667/0.714/0.938/(0.793)	0.840/0.733/0.758/0.822/(0.790)	0.938
RF	0.657	0.711/0.621/0.600/0.667/(0.652)	0.800/0.545/0.514/0.750/(0.657)	0.753/0.581/0.554/0.706/(0.652)	0.858
LR	0.650	0.689/0.621/0.630/0.641/(0.647)	0.775/0.545/0.486/0.781/(0.650)	0.729/0.581/0.548/0.704/(0.643)	0.835
GB	0.643	0.750/0.500/0.548/0.767/(0.644)	0.750/0.424/0.657/0.719/(0.643)	0.750/0.459/0.597/0.742/(0.641)	0.869
LDA	0.721	0.857/0.625/0.632/0.771/(0.726)	0.750/0.606/0.686/0.844/(0.721)	0.800/0.615/0.658/0.806/(0.722)	0.913

**Table 5:** The different classifiers' performances based on CNN feature vector selected by Lasso (60) in experiment 3.

Classifier	Accuracy	Precision (GOLD 0/I/II/III&IV (mean))	Recall (GOLD 0/I/II/III&IV (mean))	*F*1-score (GOLD 0/I/II/III&IV (mean))	AUC
SVM	0.629	0.811/0.450/0.552/0.706/(0.637)	0.750/0.545/0.457/0.750/(0.629)	0.779/0.493/0.500/0.727/(0.630)	0.880
MLP	0.821	0.919/0.722/0.833/0.811/(0.826)	0.850/0.788/0.714/0.938/(0.821)	0.883/0.754/0.769/0.870/(0.821)	0.946
RF	0.600	0.638/0.480/0.594/0.639/(0.590)	0.750/0.364/0.543/0.719/(0.600)	0.690/0.414/0.567/0.676/(0.591)	0.858
LR	0.650	0.714/0.500/0.538/0.771/(0.633)	0.875/0.455/0.400/0.844/(0.650)	0.787/0.476/0.459/0.806/(0.636)	0.866
GB	0.600	0.714/0.395/0.538/0.793/(0.613)	0.750/0.515/0.400/0.719/(0.600)	0.732/0.447/0.459/0.754/(0.602)	0.869
LDA	0.657	0.771/0.526/0.541/0.833/(0.670)	0.675/0.606/0.571/0.781/(0.657)	0.720/0.563/0.556/0.806/(0.662)	0.898

**Table 6:** The different classifiers' performances based on radiomics feature vector (1316) in experiment 4.

Classifier	Accuracy	Precision (GOLD 0/I/II/III&IV (mean))	Recall (GOLD 0/I/II/III&IV (mean))	*F*1-score (GOLD 0/I/II/III&IV (mean))	AUC
SVM	0.643	0.784/0.514/0.514/0.793/(0.655)	0.725/0.576/0.543/0.719/(0.643)	0.753/0.543/0.528/0.754/(0.647)	0.863
MLP	0.786	0.857/0.731/0.692/0.848/(0.784)	0.900/0.576/0.771/0.875/(0.786)	0.878/0.644/0.730/0.862/(0.782)	0.919
RF	0.664	0.762/0.586/0.561/0.750/(0.668)	0.800/0.515/0.657/0.656/(0.664)	0.780/0.548/0.605/0.700/(0.664)	0.886
LR	0.679	0.850/0.567/0.564/0.710/(0.680)	0.850/0.515/0.629/0.688/(0.679)	0.850/0.540/0.595/0.698/(0.678)	0.863
GB	0.729	0.795/0.724/0.690/0.684/(0.727)	0.875/0.636/0.571/0.812/(0.729)	0.833/0.677/0.625/0.743/(0.724)	0.906
LDA	0.379	0.357/0.278/0.407/0.548/(0.395)	0.250/0.455/0.314/0.531/(0.379)	0.294/0.345/0.355/0.540/(0.377)	0.639

**Table 7:** The different classifiers' performances based on the radiomics feature vector selected by Lasso (106) in experiment 4.

Classifier	Accuracy	Precision (GOLD 0/I/II/III&IV (mean))	Recall (GOLD 0/I/II/III&IV (mean))	*F*1-score (GOLD 0/I/II/III&IV (mean))	AUC
SVM	0.736	0.816/0.606/0.694/0.818/(0.737)	0.775/0.606/0.714/0.844/(0.736)	0.795/0.606/0.704/0.831/(0.736)	0.915
MLP	0.829	0.864/0.840/0.750/0.857/(0.828)	0.950/0.636/0.771/0.938/(0.829)	0.905/0.724/0.761/0.896/(0.824)	0.950
RF	0.786	0.809/0.750/0.774/0.794/(0.783)	0.950/0.636/0.686/0.844/(0.786)	0.874/0.689/0.727/0.818/(0.781)	0.928
LR	0.693	0.800/0.667/0.630/0.636/(0.689)	0.900/0.485/0.486/0.875/(0.693)	0.847/0.561/0.548/0.737/(0.680)	0.886
GB	0.736	0.766/0.708/0.686/0.765/(0.732)	0.900/0.515/0.686/0.812/(0.736)	0.828/0.596/0.686/0.788/(0.729)	0.928
LDA	0.786	0.829/0.706/0.774/0.824/(0.785)	0.850/0.727/0.686/0.875/(0.786)	0.840/0.716/0.727/0.848/(0.784)	0.920

**Table 8:** The MLP classifier's performance with different feature vectors in experiment 5.

Feature vectors	Accuracy	Precision (GOLD 0/I/II/III&IV (mean))	Recall (GOLD 0/I/II/III&IV (mean))	*F*1-score (GOLD 0/I/II/III&IV mean))	AUC
CNN feature vector selected by Lasso (60)	0.821	0.919/0.722/0.833/0.811/(0.826)	0.850/0.788/0.714/0.938/(0.821)	0.883/0.754/0.769/0.870/(0.821)	0.946
Radiomics feature vector selected by Lasso (106)	0.829	0.864/0.840/0.750/0.857/(0.828)	0.950/0.636/0.771/0.938/(0.829)	0.905/0.724/0.761/0.896/(0.824)	0.950
Combined feature vector (166)	0.879	0.905/0.885/0.861/0.861/(0.879)	0.950/0.697/0.886/0.969/(0.879)	0.927/0.780/0.873/0.912/(0.875)	0.971

**Table 9:** 3D ResNet's performance based on MLP classifier with the combined feature vector (166).

3D ResNet	Accuracy	Precision (GOLD 0/I/II/III&IV (mean))	Recall (GOLD 0/I/II/III&IV (mean))	*F*1-score (GOLD 0/I/II/III&IV (mean))	AUC
3D ResNet10	0.879	0.905/0.885/0.861/0.861/(0.879)	0.950/0.697/0.886/0.969/(0.879)	0.927/0.780/0.873/0.912/(0.875)	0.971
3D ResNet18	0.871	0.907/0.923/0.875/0.795/(0.877)	0.975/0.727/0.800/0.969/(0.871)	0.940/0.814/0.836/0.873/(0.869)	0.950
3D ResNet34	0.864	0.884/0.828/0.853/0.882/(0.862)	0.950/0.727/0.829/0.938/(0.864)	0.916/0.774/0.841/0.909/(0.862)	0.960

## Data Availability

The datasets used and analyzed during the current study are available from the corresponding authors on reasonable request.
